The article "Short-term periodic consumption of multiprobiotic from childhood improves insulin sensitivity, prevents development of non-alcoholic fatty liver disease and adiposity in adult rats with glutamate-induced obesity" was published in 2014. Journal: BMC Complement Altern Med.

# Short-term periodic consumption of multiprobiotic from childhood improves insulin sensitivity, prevents development of non-alcoholic fatty liver disease and adiposity in adult rats with glutamate-induced obesity

**DOI:** 10.1186/1472-6882-14-247

**Published:** 2014-07-16

**Authors:** Oleksandr Savcheniuk, Nazarii Kobyliak, Maryana Kondro, Oleksandr Virchenko, Tetyana Falalyeyeva, Tetyana Beregova

**Affiliations:** 1 Taras Shevchenko National University of Kyiv, Volodymyrska Str., 64/13, Kyiv 01601, Ukraine; 2 Bogomolets National Medical University, T. Shevchenko boulevard, 13, Kyiv 01601, Ukraine; 3 Danylo Halytsky Lviv National Medical University, Pekarska Str., 69, Lviv 79010, Ukraine

**Keywords:** Probiotics, Obesity, Glutamate, Leptin, Adiponectin, Insulin, Non-alcoholic fatty liver disease

## Abstract

**Background:**

Today the impairment of metabolism and obesity are being extensively investigated due to the significant increase of the prevalence of these diseases. There is scientific evidence that probiotics are beneficial for human health. Thus, the aim of the study was to investigate the effect of multiprobiotic “Symbiter acidophilic concentrated” on obesity parameters in the rats under experimental obesity.

**Methods:**

The study was carried out on 60 newborn Wistar rats, divided into 3 groups, 20 animals in each (females – n = 10, males – n = 10): intact rats, monosodium glutamate (MSG-) and MSG + probiotic group. Rats of intact group were administered with saline (8 μl/g, subcutaneously (s.c.)). Newborns rats of MSG-group and MSG + probiotic group were injected with a solution of MSG (4.0 mg/g) s.c. at 2^nd^ – 10^th^ postnatal days. The MSG + probiotic group was treated with 140 mg/kg (1.4 × 10^10^ CFU/kg) of multiprobiotic “Symbiter”. MSG-group was treated with 2.5 ml/kg of water (per os) respectively. Administration was started at the age of 4 weeks just after wean and continued for 3 month intermittently alternating two-week course of introduction with two-week course of break.

**Results:**

Neonatal treatment with MSG caused a stunted growth in both MSG-groups, which manifested with significantly smaller naso-anal length compared to adult intact rats. There was no significant difference in weight between intact and MSG-groups on 120^th^ day. The adiponectin level in the serum of rats with MSG-induced obesity decreased by 2.43 times (p = 0.001) in males and 1.75 (p = 0.020) in females. Concentration of leptin in adipose tissue were significantly higher by 45.9% (p = 0.019) and 61.2% (p = 0.009) respectively in males and females compared to intact rats. Our study has indicated that daily oral administration of multiprobiotic to neonatal MSG-treated rats by 2-week courses led to significant reduce of total body and VAT weight with subsequent improvement in insulin sensitivity and prevention of non-alcoholic fatty liver (NAFLD) development.

The article "Short-term periodic consumption of multiprobiotic from childhood improves insulin sensitivity, prevents development of non-alcoholic fatty liver disease and adiposity in adult rats with glutamate-induced obesity" was published in 2014. Journal: BMC Complement Altern Med.

**Conclusions:**

These results have shown that periodic treatment with multiprobiotic prevents the MSG-induced obesity and NAFLD development.

## Background

Obesity has dramatically increased during the past decades and has now reached epidemic proportions in both developed and developing countries [1,2]. It is a heterogeneous disorder which has been associated with an increased risk of many serious illnesses such as cardiovascular diseases [3], hypertension [4], dyslipidemia [4], diabetes mellitus [5] and some types of cancer including colon cancer [6], lung cancer [7], breast cancer [8], uterine [9] and ovarian cancer [10]. As of 2008, The World Health Organization claimed that 1.5 billion adults, in the age of 20 and older, were overweight. Among them over 200 million of men and nearly 300 million of women were obese [11]. The rate of obesity also increases with age, at least up to 50 or 60 years old [12].

Most of medications for treatment of obesity are taken out the production because of their adverse effects. Orlistat is the only drug that could be taken by patients for the prolonged time. However, little attention is paid to the search of means for obesity prophylaxis. In current scientific literature there are a lot of studies that confirm beneficial effects of probiotics on human organism. The question about probiotics impact on fat metabolism and obesity is being actively debated in the scientific literature. The gut microbiota has been recently proposed to be an environmental factor involved in the control of body weight and energy homeostasis [13-17]. This “exteriorized organ” contributes to human homeostasis via multiple metabolic functions and diverse control mechanisms.

In several studies it was revealed the positive effects of probiotics use under the conditions of experimental obesity [18,19]. In our previous work we have shown that probiotics mixture of lyophilized strains *Lactobacillus casei* IMVB-7280, *Bifidobacterium animalis* VKL and *Bifidobacterium animalis* VKB at least partially prevent the MSG-induced obesity in rats [20]. But studies have shown that multistrain probiotics are more effective than monostrain probiotics [21]. Also it is interesting to compare the influence of the lyophilized and alive strains on the obesity and reveal the gender-specific differences in the obesity development. Given the above the aim of our work was to investigate the prophylactic influence of short periodical courses of the alive multiprobiotic administration on the obesity and non-alcoholic fatty liver development (NAFLD) development induced by the neonatal MSG treatment in 4-month male and female rats.

The article "Short-term periodic consumption of multiprobiotic from childhood improves insulin sensitivity, prevents development of non-alcoholic fatty liver disease and adiposity in adult rats with glutamate-induced obesity" was published in 2014. Journal: BMC Complement Altern Med.

## Methods

### Ethics statement

This study was carried out in strict accordance with the recommendations in the Guide for the Care and Use of Laboratory Animals of the National Institutes of Health and the general ethical principles of animal experiments, approved by the First National Congress on Bioethics Ukraine (September 2001). The protocol was approved by the Committee on the Ethics of Animal Experiments of the Taras Shevchenko National University of Kyiv (Protocol number: 18/2013). The rats were kept in collective cages in controlled conditions of temperature (22 ± 3°C), light (12 h light/dark cycle) and relative humidity (60 ± 5%). The animals were fed laboratory chow (PurinaW) and tap water *ad libitum*.

### Study design

We included 60 newborn Wistar rats, divided to 3 groups of 20 animals each. All groups were equally represented by both sexes (females – n = 10, males – n = 10). Newborns rats of intact group were administered with saline subcutaneously (s.c.) in the volume of 8 μl/g at 2^nd^, 4^th^, 6^th^, 8^th^ and 10^th^ postnatal days. Newborns rats of MSG-group and MSG + probiotic group received a solution of MSG (4.0 mg/g of body weight) s.c. at 2^nd^, 4^th^, 6^th^, 8^th^ and 10^th^ postnatal days [22]. Within 4 months after birth rats were on a normal diet. MSG + probiotic group received multiprobiotic “Symbiter” in dose 140 mg/kg (1.4 × 10^10^ CFU/kg) at volume 2.5 ml/kg per os (p.o.). Multiprobiotic contains concentrated biomass of 14 probiotic bacteria of genera *Bifidobacterium*, *Lactobacillus*, *Lactococcus*, *Propionibacterium*. MSG-group respectively received 2.5 ml/kg of water (p.o.). Administration was started at the age of 4 weeks just after wean and continued for 3 month intermittently alternating two-week course of introduction with two-week course of break.

### Anthropometric measurements and obesity parameter assessment

During 4 months in all groups the changes of body weight and food intake were analyzed. In adult age, rats from three experimental groups (n = 60) were weighed and killed by cervical dislocation under urethane anesthesia. We dissected and weighed visceral adipose tissue (VAT) (epididymal, perirenal and omental fat).

For each animal at month 4 of life (120 days) we determined existence of obesity using Lee index. It was calculated as follow: the cube root of body weight (g)/nasoanal length (cm). Rats presenting values higher than 0.300 were classified as obese, equal to or less than 0.300 as normal [23].

### Sample collection and blood biochemistry analysis

Rats of all groups were fasted for approximately 12 hours prior sacrifice. Rats were sacrificed by cervical dislocation under urethane anesthesia. Blood was drawn from the apex of the cardiac ventricle and few blood drops were collected into a microcentrifuge tube containing a mixture of NaF and EDTA in a 2:1 (w/w) ratio. For blood glucose determination we used Trinder glucose oxidase method on this aliquot of blood. The remaining blood sample was collected into a sterile tube and centrifuged at 3,500 rpm (2260 g) for 15 minutes. After centrifugation serum supernatant for further analysis was aliquoted into microcentrifuge tubes and stored at -80°C. Serum insulin was determined using the Rat/Mouse Insulin ELISA Kit (Linco Research, USA). The HOMA-IR was calculated as the product of multiplying of fasting blood glucose and serum insulin divided by 22.5 [24]. ELISA was used for determination of serum adiponectin and leptin level and the VAT leptin by commercial kits «BioVendor» (Czech Republic). The VAT for measuring leptin was promptly harvested and immediately flash-frozen in liquid nitrogen and stored at -80°C. After defrosting the adipose tissue was homogenized with TES-buffer (pH = 7.4, 10 mM of tris(hydroxymethyl)aminomethane, 1 mM of EDTA, 250 mM of saccharose, inhibitors of protease (2,5 μg/ml of leupeptin, 2,5 μg/ml of aprotinin, 1 mM phenylmethanesulfonyl fluoride), 1% Triton X-100) (1:4). At next step the homogenate was centrifuged at 14000 rpm for 15 min under +4°C. The bottom layer of the supernatant was harvested for the leptin measuring.

The article "Short-term periodic consumption of multiprobiotic from childhood improves insulin sensitivity, prevents development of non-alcoholic fatty liver disease and adiposity in adult rats with glutamate-induced obesity" was published in 2014. Journal: BMC Complement Altern Med.

### Liver histology assessment

For histological analysis liver tissue samples from both the right and left hepatic lobes were taken (sample size 0.5 × 0.5 cm). After fixed for 24 hours in a liquid Buena, fragments of liver were dehydrated in alcohols of increasing concentrations (from 70 ° to 96 °), embedded in paraffin and then cut with a thickness of 5-6 microns and stained with hematoxylin-eosin. A pathologist blinded to group distributions performed the histological analyses of slides using light microscopy («Olympus», Japan). To assess morphological changes in liver we used NAS (NAFLD activity score), which includes histological features and has been defined as unweighted sum of scores for steatosis (0-3), lobular inflammation (0-3) and ballooning (0-2). Acording to NAS scores ≥5 are diagnosed as non-alcoholic steatohepatitis (NASH), and cases with a NAS <3 are mentioned as not NASH [25].

### Statistical analysis

Statistical analysis performed by using SPSS-20 software. All data in this study were expressed as means ± standard deviation (M ± SD) or %. Data distribution was analyzed using the Kolmogorov-Smirnov normality test. Continuous variables with parametric distribution were then analyzed using Analysis of Variance (ANOVA) and if the results were significant, a Fisher’s LSD Post Hoc test was performed. For data with non-parametric distribution Kruskall-Wallis test was used. Estimation of gender specific changes performed using Student’s *t* test for unpaired values. For comparisons of categorical variables we conducted χ^2^ test. The difference between groups was defined to be statistically significant when a p-value was less than 0.05.

The article "Short-term periodic consumption of multiprobiotic from childhood improves insulin sensitivity, prevents development of non-alcoholic fatty liver disease and adiposity in adult rats with glutamate-induced obesity" was published in 2014. Journal: BMC Complement Altern Med.

## Results

### Impact of probiotic short-term courses on body weight and obesity parameters

Figure 1 shows sex specific weight gain from 30 to 120 days of age in all experimental rats groups. In female rats on day 30, 60 and 90 we observed significant higher body weight in MSG- group comparative to intact control. But on day 120 the weight did no differ between intact and MSG- groups (p = 0.914). Short-term periodic administration of probiotic beginning from 30 days age lead to weight reduction by 17.3% (p = 0.001) at 120 days age in MSG-probiotic female rats comparative to MSG-group (Figure 1A). Also the body weight in this group were significantly lower by 14.3% (p = 0.001) comparative to intact rats (Figure 1A).Unlike female, in male rats on 30 days age we didn’t find significant changes in body weight at all experimental groups. Beginning from day 60 we established significant weight gain in MSG-group comparative to other groups and at day 120 the average rats body mass were 263.4 ± 26.9 g. Specifically, that additional diet correction with multiprobiotic “Symbiter” led to weight reduction by 14.5% (p = 0.005) compared to the value seen in MSG-rats after 3 month of feeding (Figure 1B).Neonatal treatment with MSG caused a stunted growth in both MSG-groups, which manifested with significant smaller naso-anal length compared to intact rats. That’s why in spite of lower weight in both sexes, after probiotic administration, we stated development of obesity in 50% of female and 40% of male animals from MSG-probiotic group compared to intact rats which was totally confirmed by Lee index higher than 0.300 (Figure 2A, B). On the other hand, short-term periodic consumption of multiprobiotic had a preventive effect on glutamate-induced obesity. Especially we observed significantly lower Lee index after probiotic correction in females (0.301 ± 0.01 vs 0.313 ± 0.01, p = 0.024) and males (0.299 ± 0.007 vs 0.319 ± 0.01, p = 0.004) compared to MSG-group (Figure 2A,B). The incidence of obesity was also higher in MSG-group – in females (90% vs 50%, p = 0,051) and respectively in males (90% vs 40%, p = 0,019).We observed 5-7 times increasing of total weight of VAT in rats with MSG-group compared to intact control (Figure 3A,B). Gender specific analysis showed the development of more pronounced visceral obesity in males, because of significant higher deposition of VAT in MSG-rats (18.72 ± 5.46 g vs 14.1 ± 2.89 g; p = 0.036).Short-term concomitant administration of probiotic bacteria led to a decrease of VAT weight by 52.43% (p = 0.001) in females and respectively by 58.86% (p = 0.001) versus MSG-group (Figure 3A, B), although its level didn’t reach the control values.Due to establish the alteration of eating behavior under conditions of MSG-induced obesity we examined food intake in one-, two-, three- and four-month rats of all group. It was shown the slight age-dependent increase in food intake both in male and female rats. We have to notice there was no any significant difference in food consumption between experimental group that suggest MSG-obesity is not a result of excessive caloric intake but associated with the metabolic disorder (Figure 4А, B ).

The article "Short-term periodic consumption of multiprobiotic from childhood improves insulin sensitivity, prevents development of non-alcoholic fatty liver disease and adiposity in adult rats with glutamate-induced obesity" was published in 2014. Journal: BMC Complement Altern Med.

**Figure 1:** **Body weight changes in rats from birth to 4-month age (M ± SD, n = 10 in each group): A –females, B – males.** * - p < 0.05 compared to intact rats, # - p < 0.05 compared to MSG-group.

**Figure 2:** **Index Lee in4-month rats (M ± SD, n = 10 in each group): A –females, B – males.** * - p < 0.05 compared to intact rats, # - p < 0.05 compared to MSG-group.

**Figure 3:** **Visceral adipose tissue weight in4-month rats (M ± SD, n = 10 in each group): A –females, B – males.** * - p < 0.05 compared to intact rats, # - p < 0.05 compared to MSG-group.

**Figure 4:** Dynamics of food intake changes in rats from 1-month to 4-month age (M ± SD, n = 10 in each group): A –females, B – males.

### Probiotic short-term courses improved insulin sensitivity in obese-induced rats

The fasting blood glucose of MSG-rats were significant higher compared to intact animals in both sexes (6.11 ± 1.15 vs 4.62 ± 0.42 mmol/L, p = 0.003 – in females; 6.17 ± 0.64 vs 4.59 ± 0.67 mmol/L, p = 0.001 – respectively in males). Female rats from MSG-probiotic group presented significant decrease of fasting glucose level by 17.34% (p = 0.024) and males – by 16.04% (p = 0.010) compared to MSG-group (Figure 5 A,B).Analysis of the HOMA-IR and serum insulin concentrations showed that under condition of MSG-induced obesity rats became insulin resistant. Both the HOMA-IR index (2.3 ± 1.2 vs 0.46 ± 0.21, p = 0.001 – in females; 2.77 ± 0.92 vs 0.66 ± 0.34, p = 0.001 – in males) and serum insulin concentration (8.19 ± 2.90 vs 2.33 ± 1.16, p = 0.001 – in females; 10.02 ± 2.62 vs 3.21 ± 1.53, p = 0.001 – in males) were significant higher in rats with MSG-induced obesity compared to control (Figures 6A,B; 7A,B). As we mentioned above the 2-week periodic multiprobiotic courses led to improvement of insulin sensitivity which manifested with significant 2-fold decrease of HOMA-IR and fasting insulinemia in relation to MSG-group. After treatment with probiotic the HOMA-IR index did not exceed the normal range, but was not significantly higher compared to intact control rats (Figure 7A, B).

The article "Short-term periodic consumption of multiprobiotic from childhood improves insulin sensitivity, prevents development of non-alcoholic fatty liver disease and adiposity in adult rats with glutamate-induced obesity" was published in 2014. Journal: BMC Complement Altern Med.

**Figure 5:** **Glucose level in serum of 4-month rats (M ± SD, n = 10 in each group): A –females, B – males.** * - p < 0.05 compared to intact rats, # - p < 0.05 compared to MSG-group.

**Figure 6:** **Insulin level in serum of 4-month rats (M ± SD, n = 10 in each group): A –females, B – males.** * - p < 0.05 compared to intact rats, # - p < 0.05 compared to MSG-group.

**Figure 7:** **HOMA-IR of 4-month rats (M ± SD, n = 10 in each group): A –females, B – males.** * - p < 0.05 compared to intact rats, # - p < 0.05 compared to MSG-group.

### Impact of short-term probiotic courses on adipocytokine levels in obese-induced rats

Analysis of the secretory function of adipose tissue showed a change in concentration adipose-derived hormones in rats with experimental obesity. Thus, the level of adiponectin in the serum of rats with MSG-induced obesity decreased by 2.43 times (p = 0.001) in males and 1.75 (p = 0.020) in females (Figure 8 A,B). Concentration of leptin in adipose tissue were higher by 45.9% (p = 0.019) and 61.2% (p = 0.009) respectively in males and females in comparison with intact control group (Figure 9A,B). In serum leptin level was lesser than in the VAT. MSG increased the leptin level by 93.3% (p < 0.05) and 83.6% (p < 0.01) respectively both in males and females (Figure 10 A,B). Gender specific analysis did not confirmed changes of leptin concentrations in adipose tissue but all experimental groups represented significantly lower serum adiponectin concentrations in males compared to females (intact – 4.29 ± 1.67 vs 6.5 ± 1.99 μg/ml, p = 0.001; MSG – 1.73 ± 0.56 vs 3.77 ± 1.64 μg/ml, p = 0.030).

**Figure 8:** **Adiponectin level in serum of 4-month rats (M ± SD, n = 10 in each group): A –females, B – males.** * - p < 0.05 compared to intact rats, # - p < 0.05 compared to MSG-group.

It was found significant increase of serum adiponectin after probiotic administration in males by 89% (p = 0.028) compared to MSG-group (Figure 8B) and females by 38.2% (p = 0.039) compared to MSG-group (Figure 8A). The VAT leptin in males decreased by 14.3% (p = 0.047) compared to MSG-group (Figure 9B) and in females – by 14.9% (p = 0.044) compared to MSG-group (Figure 9A). The serum leptin in MSG-probiotic group decreased insignificantly (Figure 10 A,B). Also showed that the concentration of adiponectin and leptin in the case of probiotics ration did not differ from the level of intact rats (Figures 7A,B; 8A,B).

The article "Short-term periodic consumption of multiprobiotic from childhood improves insulin sensitivity, prevents development of non-alcoholic fatty liver disease and adiposity in adult rats with glutamate-induced obesity" was published in 2014. Journal: BMC Complement Altern Med.

**Figure 9:** **Leptin level in adipose tissue of 4-month rats (M ± SD, n = 10 in each group): A –females, B – males.** * - p < 0.05 compared to intact rats, # - p < 0.05 compared to MSG-group.

**Figure 10:** **Leptin level in serum of 4-month rats (M ± SD, n = 10 in each group): A –females, B – males.** * - p < 0.05, p < 0.01 compared to intact rats.

Thus, intermittent administration of probiotics for two weeks courses restored the hormonal activity of adipose tissue.

### Morphological changes in rat liver under the conditions of obesity and probiotic administration

We found significantly lower total score (0.95 ± 0.15 vs 3.3 ± 0.28, p < 0.001), degree of steatosis (0.85 ± 0.13 vs 2.15 ± 0.16, p < 0.001) and manifestation of lobular inflammation (0.1 ± 0.06 vs 0.95 ± 0.15, p < 0.001) due to NAFLD activity score in MSG-probiotic group compared to MSG-obesity (Table 1).

**Table 1:** Morphological changes in rats liver assessed by NAFLD activity score (NAS)

	**Intact group (n = 20)**	**MSG-obesity (n = 20)**	**MSG-probiotic (n = 20)**
Steatosis (0-3)	0.10 ± 0.1^a^	2.15 ± 0.16^b^	0.85 ± 0.13^c^
Lobular inflammation (0-2)	0.0 ± 0.0^a^	0.95 ± 0.15^b^	0.1 ± 0.06^a^
Ballooning degeneration (0–2)	0.0 ± 0.0^a^	0.15 ± 0.08^a^	0.0 ± 0.0^a^
Total NAS (0–8)	0.10 ± 0.1^a^	3.3 ± 0.28^b^	0.95 ± 0.15^c^

Data are presented as the M ± SEM. One-way ANOVA with post hoc comparisons by Fisher LSD test were performed for data analysis. ^a^, ^b^, ^c^: shows significant differences in the same row (p < 0.05).

## Discussion

A lot of factors lead to development of obesity. The most important factors contributing to fat accumulation are widespread net of fast food restaurants, which offer the variety of energy-dense foods and low physical activity and the genetic inheritance. Also It was shown contributing of microorganisms, increasing maternal age, greater fecundity among people with higher adiposity, sleep debt, endocrine disruptors, pharmaceutical iatrogenesis, reduction in variability of ambient temperatures and intrauterine effects to the obesity [26,27]. In general obesity develops when the body receives more energy with food than it can spend. Not the least role in increased energy consumption plays monosodium glutamate (C_5_H_8_NO_4_Na, MSG, E621) which is food additive and is found especially in fast food.

MSG can be formed naturally in various foods (cheese, meat, etc.) [28]. Also it is largely used in the food industry because it improves the taste of food and even can mask the bad taste of stale products. That is why its consumption steadily increases worldwide. In 1968, a report appeared in the New England Journal of Medicine, describing a complex of symptoms in patients who dined in Chinese restaurants. The symptoms of the so-called «Chinese restaurant syndrome» included numbness, radiating to the back, arms, and neck; weakness; and palpitations [29]. Cross-sectional and longitudinal studies in healthy Chinese subjects showed correlation of MSG intake with an increased risk of being overweight irrespective of the total calorie intake and physical activity [30,31].

The article "Short-term periodic consumption of multiprobiotic from childhood improves insulin sensitivity, prevents development of non-alcoholic fatty liver disease and adiposity in adult rats with glutamate-induced obesity" was published in 2014. Journal: BMC Complement Altern Med.

Animal models support a causative association between obesity and neonatal or maternal administration of high doses of MSG [32]. MSG acts on immature neurological mechanisms that regulate food intake and energy expenditure by ablating cells in the arcuate nucleus of the hypothalamus and destroying circumventricular neurons. MSG altered the production of orexigenic and anorexigenic molecules as proopiomelanocortin, cocaine- and amphetamine-regulated transcript and neuropeptide Y [33]. Neonatal neurotoxity effect of MSG leading to the development of neurochemical, endocrine, metabolic and behavioural abnormalities in adulthood including hypophagia, obesity, hypoactivity, delayed puberty, and elevated plasma corticosterone levels [34]. Furthermore, stunted growth, increased adipose tissue stores, and a marked increase in plasma triglycerides [35], insulin [36] and fasting glucose levels [37] have been noted in rats.

Most of medications for treatment of obesity are taken out the production because of their adverse effects. Orlistat is the only drug that could be taken by patients for the prolonged time. However, little attention is paid to the search of means for prophylaxis of obesity. In current scientific literature there are a lot of studies that confirm beneficial effects of probiotics on human organism. The question about probiotics impact on fat metabolism and obesity is being actively debated in the scientific literature. The gut microbiota has been recently proposed to be an environmental factor involved in the control of body weight and energy homeostasis [13-17]. This “exteriorized organ” contributes to our homeostasis via multiple metabolic functions and diverse control mechanisms. For example it involved in the extraction of calories from ingested dietary substances, and it helps to store these calories in host adipose tissue for later use. Pioneers in study of the gut microbiota role for the development of obesity and fat mass storage were Gordon et al. They determined that parallel with lower energy intake young conventionally reared mice had higher on 42% and 47% total body fat and gonadal fat mass respectively as compared with germ-free mice [25]. Authors firstly declared that microbiota itself can increase energy yield from diet of the host organism’s. Colonization within two weeks of young germ-free mice with microbiota from conventionally reared mice is associated with increased insulin resistance and provokes a 60% increase in total body fat mass despite lower energy intake [13]. This fat mass gain was even more pronounced when the gut microbial community was derived from genetically obese (*ob/ob*) mice [17].

The article "Short-term periodic consumption of multiprobiotic from childhood improves insulin sensitivity, prevents development of non-alcoholic fatty liver disease and adiposity in adult rats with glutamate-induced obesity" was published in 2014. Journal: BMC Complement Altern Med.

Gut microbiota may change with body weight. Ley et al. [27] recently analysed 5,088 bacterial 16S rRNA gene sequences from the distal intestinal (cecal) microbiota of genetically obese ob/ob mice, lean ob/+and wild-type siblings, and their ob/+mothers, all fed the same polysaccharide-rich diet. They demonstrated that compared with lean mice obese animals have a 50% reduction in the abundance of Bacteroidetes and a proportional increase in Firmicutes. Feeding of a high-fat/high-polysaccharide diet to genetically wild-type rodents led to similar microbial changes [16]. Methanogenic Archaea also located in ob/ob mice, which lead to increasing of the efficiency of bacterial fermentation [29].

Similar to these animal experiments, Ley et al. demonstrated that the ratio of *Firmicutes/Bacteroidetes* in the distal gut microbiota is also increase in obese people by comparison with lean people [38]. This proportion increases with weight loss on a fat-restricted or carbohydrate-restricted diet. Another study, without limit of dietary components, described that *Prevotellaceae*, a subgroup of *Bacteroidetes*, are significantly enriched in obesity and demonstrated that *Firmicutes* are dominant in lean and obese individuals [39]. The differences in microbial composition between two studies were explained by an increased capacity of the obesity-associated microbiome to harvest energy from the diet.

Controversial data were recently reported by Schwiertz and colleagues [40]. They determined lower ratios of *Firmicutes* to *Bacterodetes* in overweight human adults compared to lean controls. Another study, using weight loss diets, found no proof of the link between the proportion of *Bacteroidetes* and *Firmicutes* and human obesity [41].

Kalliomaki et al. [42] examined if early differences in gut microbiota composition in children can guide weight development throughout early childhood. Overweight and obese children (n = 25) were selected. Early fecal microbiota composition was analyzed by fluorescent in situ hybridization (FISH) with additional flow cytometry. They find that bifidobacterial numbers in fecal samples during infancy were higher in children remaining normal weight than in children becoming overweight, [2.19 × 10^9^ [1.10–5.28] cells/g vs 1.20 × 10^9^ [0.48–1.59] cells/g; p = 0.02]. Overweight was also associated with a greater number of Staphylococcus aureus. Author suggested that changes in early life gut microbiota composition may be associated with an increased risk of developing obesity in later life.

The article "Short-term periodic consumption of multiprobiotic from childhood improves insulin sensitivity, prevents development of non-alcoholic fatty liver disease and adiposity in adult rats with glutamate-induced obesity" was published in 2014. Journal: BMC Complement Altern Med.

These data suggest an association between obesity and the intestinal microbiota. In several studies it was revealed the positive effects of probiotics use under the conditions of experimental obesity [18,19]. In our previous work we have shown that probiotics mixture of lyophilized strains *Lactobacillus casei* IMVB-7280, *Bifidobacterium animalis* VKL and *Bifidobacterium animalis* VKB at least partially prevent the MSG-induced obesity in rats [20]. But studies have shown that multistrain probiotics are more effective than monostrain probiotics [21]. Also it is interesting to compare the influence of the lyophilized and alive strains on the obesity and reveal the gender-specific differences in the obesity development. Given the above the aim of our work was to investigate the prophylactic influence of short periodical courses of the alive multiprobiotic administration on the obesity development induced by the neonatal MSG treatment in 4-month male and female rats.

Thus, finding new non-toxic means of prevention and treatment of obesity is one of the major problems of modern science. Our study showed that short-term periodic administration of multiprobiotic beginning from childhood prevented development of MSG-induced obesity in adult rats. This was confirmed by significant lower incidence of obesity and mean value for Lee index and reduction of total body and VAT weight in rats after correction with multiprobiotic “Symbiter” compared to MSG-group.

The most frequent cause which leads to the obesity development is a dysbalance between energy intake and energy expenditure. In this complex process genetic susceptibility, environmental and lifestyle factors are involved. Recent advances in next generation sequencing technology and mechanistic testing in gnotobiotic mice have identified the gut microbiota as an environmental factor that increase energy yield from diet, regulate metabolism, integrate peripheral and central food intake regulatory signals and thereby increase body weight. Underlying mechanisms whereby the gut microbiota contributes to host metabolism were revealed from studies on germ-free mice which were protected against developing diet-induced obesity.

One of the key mechanism by which germ-free animals seem protected from diet-induced obesity is elevated levels of fasting-induced adipose factor (FIAF), also known as angiopoietin-like protein 4. FIAF is a circulating lipoprotein lipase (Lpl) inhibitor produced by the intestine, liver and adipose tissue [43]. Conventionalization of germ-free mice suppresses expression of *Fiaf* in gut epithelial cells [13]. Thereby lead to higher adipocyte Lpl activity results in increased cellular uptake of fatty acids, adipocyte triglyceride accumulation and greater fat storage. Germ-free *Fiaf–/–* mice are similarly obese to their conventionally reared counterparts. After conventionalization germ-free *Fiaf–/–* mice produced higher on 57% total body fat as observed in wild-type littermates [13]. Consistently, germ-free *Fiaf–/–* mice fed by high-fat, high-carbohydrate diet were not protected from diet-induced obesity, suggesting that FIAF is a mediator of microbial regulation of energy storage [44].

The article "Short-term periodic consumption of multiprobiotic from childhood improves insulin sensitivity, prevents development of non-alcoholic fatty liver disease and adiposity in adult rats with glutamate-induced obesity" was published in 2014. Journal: BMC Complement Altern Med.

In contrast, mice fed by high-fat diet complemented with *Lactobacillus paracasei* exhibited significantly reduced body fat, which was paralleled by increased circulating levels of FIAF [45]. Fleissner et al. showed that germ-free mice on high-fat diet showed increased intestinal mRNA expression of *Fiaf* with no major changes in circulating FIAF compared with conventionalised mice, suggesting that FIAF mechanism is not universally associated with gut microbiota-related fat mass development [46].

Furthermore, Backhed and colleagues have also demonstrated that germ-free mice have increased levels of phosphorylated AMP-activated protein kinase (AMPK) in muscle and liver. AMPK is a key enzyme that controls cellular energy status which activates key enzymes of mitochondrial fatty acid oxidation, including acetyl-CoA carboxylase (ACC) and carnitine-palmitoyltransferase I (CTP1), indicative of increased energy expenditure. The exact pathway whereby the microbiota signals to liver or skeletal muscle AMPK is unclear but appears to be independent from FIAF [44].

Another mechanism is related to energy extraction from undigested food components. The gut microbiota that digest complex dietary carbohydrates produces many monosaccharides and short-chain fatty acids (SCFAs) such as acetate, propionate, and butyrate [44] which represent an important energy source. Conventionalization of germ-free mice doubled the density of small intestinal villi capillaries [47] and enhanced uptake of this components from the gut into the portal blood and eventually participate in hepatic de novo lipogenesis promoting fat accumulation in the liver and adipose tissue [44]. This reaction controlled by carbohydrate responsive element binding protein (ChREBP) and sterol responsive element binding protein (SREBP-1) [48]. We observed that multiprobiotic administration from childhood lead to histological features improvement which manifested with hepatic steatosis attenuation and decreased lobular inflammation in MSG-probiotic group. NASH we confirmed only in 20% of rats with MSG-obesity (p = 0.035).

The article "Short-term periodic consumption of multiprobiotic from childhood improves insulin sensitivity, prevents development of non-alcoholic fatty liver disease and adiposity in adult rats with glutamate-induced obesity" was published in 2014. Journal: BMC Complement Altern Med.

SCFAs act in the gut as signaling molecules and are specific ligands for at least two G protein-coupled receptors, GPR41 and GPR43, mainly expressed by intestinal epithelial cells [49,50]. Samuel et al. have demonstrated that conventionally raised *Gpr41*–/– mice and germ-free *Gpr41–/–* mice colonized with only *Bacteroides thetaiotaomicron* and *Methanobrevibacter smithii* are significantly leaner than wild-type littermates, while there are no differences between wild-type or *Gpr41–/–* germ-free mice [51]. Gpr41, which is produced by enteroendocrine cells, might be a regulator of host energy balance through effects that are dependent upon the gut microbiota. Activation of GPR41 increases production of peptide YY (PYY), an enteroendocrine cell hormone that normally inhibits gut motility, increases intestinal transit rate and reduces extraction of energy from the diet, thus affecting peripheral glucose utilisation [51]. Recent study has shown that *Gpr43–/–* mice are resistant to diet-induced obesity and insulin resistance, at least partly due to Gpr43-regulated energy expenditure [52].

Some lines of experimental evidence suggest that high-fat diets may affect epithelial integrity due to changes in the distribution and localisation of Zonula Occludens-1 (ZO-1) and Occludin (two tight junction proteins) in intestinal tissue and hence lead to impaired gut permeability, and consequently to low-grade systemic inflammation [53-55]. Cani et al. demonstrated that bacterial lipopolysaccharide (LPS), which continuously produced in the gut through lysis of gram-negative bacteria is a microbiota-related factor which can trigger the inflammatory process by binding to the CD14 toll-like receptor-4 (TLR-4) complex at the surface of innate immune cells [55]. Author mentioned that after 4 weeks of high-fat feeding, mice exhibited an obese phenotype accompanied by a change in gut microbiota composition (the reduction of Bifidobacteria and Eubacteria spp.) and a two- to threefold increase in circulating LPS levels, which they called “metabolic endotoxemia” since LPS plasma concentrations were much lower than those observed during septic shock [56]. In fact, in this study, continuous subcutaneous low-rate infusion of LPS led to excessive weight gain and insulin resistance in mice. Moreover, LPS receptor *Cd14-/-* mice tend to be resistant to this chronic inflammatory state and were hypersensitive to insulin even when they were fed a normal diet, suggesting that CD14 may modulate insulin sensitivity in physiological conditions [57]. Deletion of TLR-4 prevented the high-fat diet–induced insulin resistance [58].

The article "Short-term periodic consumption of multiprobiotic from childhood improves insulin sensitivity, prevents development of non-alcoholic fatty liver disease and adiposity in adult rats with glutamate-induced obesity" was published in 2014. Journal: BMC Complement Altern Med.

They also demonstrated that modulation of gut microbiota, e.g. by antibiotic treatment or dietary intervention with oligofructoses, reduced metabolic endotoxemia and the cecal content of LPS, improved glucose intolerance, insulin sensitivity and decreased body weight gain in both high-fat fed and *ob/ob* mice [59,60].

In models of diabetes, probiotic intervention has been examined for its ability to impact on metabolic biomarkers of disease. Tabuchi et al showed that *Lactobacillus rhamnosus* GG improved glucose tolerance in the streptozotocin-induced rat model of diabetes possibly due to prevention of a decrease in insulin secretion [61]. Studies using the traditional Indian yoghurt – dahi supplemented with probiotic strains of *Lactobacillus acidophilus* and *L. casei* have shown that this product can improve markers of diabetes, including hyperglycemia, hyperinsulinemia in high-fructose induced rat models of diabetes [62,63].

We first studied influence of probiotic administration for insulin sensitivity in rat model of MSG-induced obesity. Nagata et al. found that mice after neonatal treatment with MSG were observed to be obese but had no polyphagia, and were glycosuric by 29 weeks of age. The pathological study showed hypertrophy of the pancreatic islet, with elevation of glucose and insulin serum concentrations at 29 and 54 weeks aged compared to control mice [32]. From the other hand in the early phase of obesity level of plasma glucose can be normal but associated with hyperinsulinemia [64] which indicates that insulin resistance is present and high insulin levels may be compensatory due to direct hypersecretion of β cells [65].

Our data is agreed with recently reported studies [62,63] and showed that in addition to reduction in total body weight administration of multiprobiotic by short courses led to improvement of insulin sensitivity that was confirmed by significant decreasing of hyperinsulinemia and HOMA-IR in MSG-probiotic group compared to MSG-animals. From the other hand we observed significant increase of serum adiponectin, which define as one of the main regulators of peripheral tissues sensitivity to insulin [66], only in females compared to MSG-group.

As previously reported for MSG rats and mice, leptin mRNA expression levels and serum levels in MSG-treated mice were significantly higher compared to that in normal controls [67,68]. The increased leptin production in adipose tissues due to pancreatic hypertrophy and hyperinsulinaemia have been reported to induce the development of leptin resistance [69]. We mentioned that probiotics helped to restore the hormonal activity of adipose tissue. Thus, concentration of leptin under the probiotics admistration did not differ from the level of intact rats.

The article "Short-term periodic consumption of multiprobiotic from childhood improves insulin sensitivity, prevents development of non-alcoholic fatty liver disease and adiposity in adult rats with glutamate-induced obesity" was published in 2014. Journal: BMC Complement Altern Med.

## Conclusion

In summary, we studied effectiveness of short-term periodic consumption of multiprobiotic from childhood on metabolic profile in adult rats with MSG-induced model of obesity. Subcutaneous neonatal injection of MSG is able to induce obesity without hyperphagia, which diagnosed by high Lee index and characterized by small corporal weight and naso-anal length. Obesity in rats caused by alterations in hypothalamic arcuate nucleus and impairs leptin and insulin signaling in this region resulting in hyperleptinemia and hyperinsulinemia.

Our study has indicated that daily oral administration of 2.5 ml/kg of alive multiprobiotic “Symbiter” containing concentrated biomass of 14 probiotic bacteria of *Bifidobacterium*, *Lactobacillus*, *Lactococcus*, *Propionibacterium* genera to neonatal MSG-treated rats by 2-weeks courses led to significant reduce of total body and VAT weight, together with improvement in insulin sensitivity and prevention of NAFLD development.

## Abbreviations

AMPK: AMP-activated protein kinase; ACC: Acetyl-CoA carboxylase; ChREBP: Carbohydrate responsive element binding protein; CTP1: Carnitine-palmitoyltransferase 1; FIAF: Fasting-induced adipose factor; FISH: Fluorescent in situ hybridization; GPR: G protein-coupled receptors; LPS: Lipopolysaccharide; Lpl: Lipoprotein lipase; NAFLD: Non-alcoholic fatty liver disease; NASH: Non-alcoholic steatohepatitis; SREBP-1: Sterol responsive element binding protein; SCFAs: Short-chain fatty acids; TLR-4: Toll-like receptor-4; VAT: Visceral adipose tissue.

## Competing interests

The authors declare to have no competing interests.

## Authors’ contributions

TB, TF and NK designed the study. OV develop the protocol and wrote the first and second drafts of the manuscript. OS performed the experimental works. MK involved in the collection of literature, interpret the results and performed the statistical analysis. All authors read and approved the final manuscript.

## Authors’ information

OS - PhD student, SRL ‘Pharmacology and Experimental Pathology’, Department of Biological and Biomedical Technology, ESC ‘Institute of Biology’, Taras Shevchenko National University of Kyiv.

NK – PhD, assistant of Endocrinology Department, Bogomolets National Medical University.

OV - PhD student, SRL ‘Pharmacology and Experimental Pathology’, Department of Biological and Biomedical Technology, ESC ‘Institute of Biology’, Taras Shevchenko National University of Kyiv.

The article "Short-term periodic consumption of multiprobiotic from childhood improves insulin sensitivity, prevents development of non-alcoholic fatty liver disease and adiposity in adult rats with glutamate-induced obesity" was published in 2014. Journal: BMC Complement Altern Med.

FT - Ph.D., D.Sci., researcher of RL “Pharmacology and Experimental Pathology” Department of Biological and Biomedical Technology ESC «Institute of Biology» Taras Shevchenko National University of Kyiv.

MK – PhD, Assosiate Professor of Department of Normal Physiology Danylo Halytsky Lviv National Medical University.

TB - Professor, Ph.D., D.Sci., SRL ‘Pharmacology and Experimental Pathology’, Department of Biological and Biomedical Technology, ESC ‘Institute of Biology’, Taras Shevchenko National University of Kyiv.

## Pre-publication history

The pre-publication history for this paper can be accessed here:

http://www.biomedcentral.com/1472-6882/14/247/prepub
